# Single Neuron for Solving XOR like Nonlinear Problems

**DOI:** 10.1155/2022/9097868

**Published:** 2022-04-28

**Authors:** Ashutosh Mishra, Jaekwang Cha, Shiho Kim

**Affiliations:** School of Integrated Technology, YICT, Yonsei University, Seoul, Republic of Korea

## Abstract

XOR is a special nonlinear problem in artificial intelligence (AI) that resembles multiple real-world nonlinear data distributions. A multiplicative neuron model can solve these problems. However, the multiplicative model has the indigenous problem of backpropagation for densely distributed XOR problems and higher dimensional parity problems. To overcome this issue, we have proposed an enhanced translated multiplicative single neuron model. It can provide desired tessellation surface. We have considered an adaptable scaling factor associated with each input in our proposed model. It helps in achieving optimal scaling factor value for higher dimensional input. The efficacy of the proposed model has been tested by randomly increasing input dimensions for XOR-type data distribution. The proposed model has crisply classified even higher dimensional input in their respective class. Also, the computational complexity is the same as that of the previous multiplicative neuron model. It has shown more than an 80% reduction in absolute loss as compared to the previous neuron model in similar experimental conditions. Therefore, it can be considered as a generalized artificial model (single neuron) with the capability of solving XOR-like real problems.

## 1. Introduction

Minski and Perpert deduced that the XOR problem requires more than one hyperplane [1]. They provide a more generalized artificial neuron model by introducing the concept of weights and proved the inability of a single perceptron for solving ‘Exclusive-OR (XOR)' [2]. The XOR problem is symmetrical to other popular and real-world problems such as XOR type nonlinear data distribution in two classes, *N*-bit parity problems. [3]. Therefore, many researchers tried to find a suitable way out to solve the XOR problem [4–15]. Although, most of the solutions are for the classical XOR problem. They either use more than one layer or provide a complex solution for two-bit logical XOR only. Few of these used the complex value neuron model, eventually creating one more layer (i.e., hidden layer). Because the complex value neuron model requires representing the real input in a complex domain, one approach is based on the multiplicative neuron model. This is translated multiplicative neuron (*π*_t_-neuron) approach [16, 17]. They have modified the *π*-neuron model (which generates the decision surfaces centered at the origin of input) to an extended multiplicative neuron, i.e., a *π*_t_-neuron model for solving the *N*-bit parity problems by creating tessellation surfaces. However, it has limitations for higher dimensional *N*-bit parity problems. It is suitable for up to six dimensions. For seven and higher dimensional inputs, it has reported poor accuracy [17]. In other words, it has a convergence problem for higher dimensional inputs. It is merely because of the multiplicative nature of the model. More clearly, the infinitesimal errors in the model obtain a much smaller value after getting multiplied in case of higher dimensional inputs, consequently vanishing the gradient. Therefore, a convergence problem occurs in this model for higher-dimensional inputs.

To overcome the issue of the *π*_*t*_-neuron model, we have proposed an enhanced translated multiplicative model neuron (*π*_*t*_-neuron) model in this paper. It helps in achieving mutually orthogonal separation in the case of two-bit classical XOR data distribution. Also, the proposed model has shown the capability for solving the higher-order *N*-bit parity problems. Therefore, it is a generalized artificial model for solving real XOR problems. To examine this claim, we have tested our model on different XOR data distributions and *N*-bit parity problems. For parity problems, we have varied the input dimension for a higher dimensional dataset. Our proposed model has no vanishing gradient issues and convergence issues for higher dimensional inputs. The proposed model has accurately classified the considered dataset.  Table 1 presents the list of variables used in this article with their meaning.

## 2. Understanding the XOR Problem

XOR is a classical problem in the artificial neural network (ANN) [18]. The digital two-input XOR problem is represented in Figure 1. By considering each input as one dimension and mapping the digital digit ‘*0*' as the negative axis and ‘*1*' as the positive axis, the same two-digit XOR problem becomes XOR type nonlinear data distribution in two-dimensional space. It is obvious here that the classes in two-dimensional XOR data distribution are the areas formed by two of the axes ‘*X*_*1*_' and ‘*X*_*2*_' (Here, *X*_*1*_ is input *1*, and *X*_*2*_ is input *2*). Furthermore, these areas represent respective classes simply by their sign (i.e., negative area corresponds to class *1*, positive area corresponds to class *2*).

There are many other nonlinear data distributions resembling XOR. *N*-bit parity problem is one such typical example. Both these problems are popular in the AI research domain and require a generalized single neuron model to solve them. We have seen that these problems require a model which can distinguish between positive and negative quantities. Interestingly, addition cannot easily separate positive and negative quantities, whereas multiplication has the basic property to distinguish between positive and negative quantities. Therefore, previous researchers suggested using a multiplicative neuron model for solving XOR and similar problems.

## 3. Translated Multiplicative Neuron (Π_*T*_-NEURON) Model

The idea of the multiplicative neuron model was initiated by Durbin et al. in 1989 [19]. They named this model the ‘*Product Units (PUs)*' and used this model to deal with the generalized polynomial terms in the input. It can learn higher-order inputs easily as compared to the additive units. This is because of its increased information capacity as compared to the additive units [19]. Though, PU has shown the capability for *N*-bit parity problems. However, it has issues in training with the standard backpropagation (BP) algorithm especially for higher-order inputs (more than three-dimensional input) [20]. According to Leerink et al., it is because of nonglobal minima trapping in the case of higher dimensional inputs [20]. Later, in 2004, Iyoda et al. proposed a single neuron based on a multiplicative neuron model, aka *π*_*t*_-neuron model, to solve the XOR and parity bit problems [16, 17]. They have modified the previous multiplicative *π*-neuron model to find a suitable tessellation decision surface. They incorporated a scaling factor, a threshold value, and used the sigmoid as an activation function to solve the *N*-bit parity problems using a single translated multiplicative neuron (the model is defined by equations (1) and (2)) [16].

(1) $$\begin{array}{c} v_{\pi -t}=b_{\pi -t}\times \prod_{i=1}^{N}\left(x_{i}-t_{i}\right);Here,{\left(b_{\pi -t}\right)}_{i}\in \mathbb{R},t_{i}\in \mathrm{\mathbb{R},} \end{array}$$

(2) $$\begin{array}{c} y=f\left(v_{\pi -t}\right). \end{array}$$

Here, ‘*v*_*π*‒t_' represents the *π*_*t*_-neuron model mathematically, ‘*y*' is the final output through the activation function ‘*f*', ‘*b*_*π‒t*_' is scaling factor, and ‘*t*_*i*_' represent the coordinates of the center of the decision surfaces [16]. Mathematically, Iyoda et al. have shown the capability of the model for solving the logical XOR and *N*-bit parity problems for ∀ *N* ≥ 1. However, this model also has a similar issue in training for higher-order inputs.

### 3.1. Limitations of Translated Multiplicative Neuron

The *π*_*t*_-neuron model has shown the appropriate research direction for solving the logical XOR and *N*-bit parity problems [16]. The reported success ratio is ‘1' for two-bit to six-bit inputs in [17]. However, in the case of seven-bit input, the reported success ratio is ‘0.6' only. Success ratio has been calculated by considering averaged values over ten simulations [17]. Also, for successful training in the case of seven-bit, it requires adjusting the trainable parameter (scaling factor *b*_*π‒t*_) [17]. This is also indicating the training issue in the case of higher dimensional inputs. Moreover, Iyoda et al. have suggested increasing the range of initialization for scaling factors in case of a seven-bit parity problem [17]. Although, after the suggested increment as well, the reported success ratio is ‘0.6' only [17]. It indicates the problem of training in the *π*_*t*_-neuron model for higher dimensional input.

### 3.2. Causes of Failure in Π_*t*_-NEURON Model

In the backpropagation algorithm, the local gradient ‘*δ*(*n*)' accounts for the required changes in the trainable parameter at ‘*n*^*th*^' iteration to obtain desired output [21]. It is equal to the product of the corresponding error signal for that neuron and the derivative of the associated activation function [21]. Backpropagation requires that the activation function should be bounded, continuous, and monotonic. Also, it should be continuously differentiable for the entire domain of the input to get optimization [22]. Sigmoid activation function ‘*ϕ*(*x*)' is preferred in the classification problem because it has met all of the aforementioned requirements [23]. Also, it is an appropriate activation function for training multiplicative neuron models [23]. Iyoda et al. have demonstrated the error gradient (∇*Ɛ*) associated with the *π*_*t*_-neuron model [17]. Here, ‘*Ɛ*(*n*)' is the error energy, i.e., the instantaneous sum of the error squares at ‘*n*^*th*^' iteration. The error gradient has two components, one is due to the scaling factor ‘(*b*_*π‒t*_),' given by equation (3), and the other is due to the thresholds ‘*t*_*i*_', given by equation (4) [17].

(3) $$\begin{array}{c} \frac{\partial \varepsilon \left(n\right)}{\partial b_{\pi -t}\left(n\right)}=\delta \left(n\right)\times \prod \left(x_{k}\left(n\right)-t_{k}\left(n\right)\right), \end{array}$$

(4) $$\begin{array}{c} \frac{\partial \varepsilon \left(n\right)}{\partial t_{i}\left(n\right)}=-\delta \left(n\right)\times b_{\pi -t}\times \prod \left(x_{k}\left(n\right)-t_{k}\left(n\right)\right);\forall \left(\text{i}\neq k\right), \end{array}$$

(5) $$\begin{array}{c} \delta \left(n\right)=e\left(n\right)\times \phi^{\prime }\left(v_{\pi -t}\left(n\right)\right). \end{array}$$

Here, ‘*n*' represents ‘*n*^*th*^' iteration, ∀ (*k* = *1*, *2*, *3*,…, *N*). ‘*x*_*k*_(*n*)' is the ‘*k*^*th*^' input for ‘*n*^*th*^' iteration, and ‘*v*_*π*‒t_(*n*)' represents *π*_*t*_-neuron model. Therefore, the error's gradient obtains a much smaller value after getting multiplied for higher dimensional inputs and becomes an infinitesimally small value. Consequently, vanishing the gradient. Therefore, a convergence problem occurs in this model.

It is inferred from Figure 1 and equation (1) that the *π*_*t*_-neuron model has ranged between [‒1, 1] for XOR and *N*-bit parity problems. Here, ‘*‒1*' corresponds to digit ‘*0*', and ‘*+1*' corresponds to digit ‘*1*'. Sigmoid function has a basic issue of vanishing gradient near the extremes as shown in Figure 2(a). However, about the XOR and *N*-bit parity problems, the input varies between [‒1, 1] only, as explained earlier. Therefore, the main region of interest is incorporated by a rectangular box of sigmoid activation function in Figure 2. Here, it is important to notice that margin between two points has been reduced by the sigmoid activation function (as shown in Figure 2(a), *ϕ* (‒1) = 0.2689, and *ϕ* (1) = 0.7311). Therefore, it leads to the smaller local gradient ‘*δ*(*n*)' value (given by Equation (5)) which consequently results in smaller error gradients (given equations (3)–(5)), eventually leading to the gradient vanishing problem.

For higher dimensional input, the error gradient (∇*Ɛ*) attains further smaller values because of the presence of the factor (∏ (*x*_*k*_(*n*) + *t*_*k*_(*n*))) in the expression of error gradients (as given by equations (3)–(5)). Therefore, the possibilities of nonconvergence/nonglobal minima problems occur in the previous *π*_*t*_-neuron model. To overcome this issue, the model should have a larger margin for the extreme values. It is possible by introducing a compensatory scaling factor in the model. It eventually scales the sigmoid activation function, as depicted in Figure 2(b). Therefore, in [17], the author suggested using a scaling factor ‘*b*_*π‒t*_'. However, it requires an optimized value of the scaling factor to mitigate the effect of multiplication and sigmoid function in higher-dimensional problems. Because the effect of multiplication and sigmoid function is severe in higher-order input, Iyoda et al. recommended initializing the scaling factor only with higher values (not to the threshold factor) for the seven-bit parity problem [17]. Convergence is not possible with a smaller scaling factor for the higher dimensional problem (results given in ‘Table 2' of [17] follow this statement). Though, the idea of increasing the learning rate for the scaling factor is worth overcoming the vanishing gradient problem in higher dimensional input. However, an optimized value of the learning rate is not suggested in the previous *π*_*t*_-neuron model. Also, it is difficult to adjust the appropriate learning rate or range of initialization of scaling factors for variable input dimensions. Therefore, a generalized solution is still required to solve these issues of the previous model. In this paper, we have suggested a generalized model for solving the XOR and higher-order parity problems by enhancing the *p*_t_-neuron model.

## 4. Related Works

Robotics, parity problems, and nonlinear time-series prediction are some of the significant problems suggested by the previous researchers where multiplicative neurons are applied. Forecasting involving the time series has been performed using the multiplicative neuron models [24–26]. Yildirim et al. have proposed a threshold single multiplicative neuron model for time series prediction [24]. They utilized a threshold value and used the particle swarm optimization (PSO) and harmony search algorithm (HSA) to obtain the optimum weight, bias, and threshold values. In [25], Yolcu et al. have used autoregressive coefficients to predict the weights and biases for time series modeling. A recurrent multiplicative neuron model was presented in [26] for forecasting time series.

Yadav et al. have also used a single multiplicative neuron model for time series prediction problems [27]. In [28], authors have used the multiplicative neuron model for the prediction of terrain profiles for both air and ground vehicles. Egrioglu et al. have represented forecasting purposes like classical time series forecasting using a single multiplicative neuron model in [29]. In [30], Gao et al. proposed a dendritic neuron model to overcome the limitation of traditional ANNs. It has utilized the nonlinearity of synapses to improve the capability of artificial neurons. A few other recent works are suggested in [31–35].

## 5. Enhanced Translated Multiplicative Neuron

We have seen the problems associated with the *π*_*t*_-neuron model. It has an issue with BP training in case of highly dense XOR data distribution and higher dimensional parity problems. In this paper, we have proposed an enhanced translated multiplicative single neuron model which can easily learn the nonlinear problems such as XOR and *N*-bit parity without any training limitations. We have modified the existing *π*_*t*_-neuron to overcome its limitations. The proposed enhanced translated multiplicative neuron model is represented in Figure 3 and described as follows:

(6) $$\begin{array}{c} v={\left(-1\right)}^{N+1}\times \prod_{i=1}^{N}\left\{\left(b_{i}\right)\times \left(x_{i}+t_{i}\right)\right\},\\ Forb_{1}=b_{2}=\cdots =b_{i}=\cdots =b;and,b\in \mathbb{R},then: \end{array}$$

(7) $$\begin{array}{c} v={\left(-1\right)}^{N+1}\times \overset{N}{\underset{i=1}{\prod }}\left\{\left(b\right)\times \left(x_{i}+t_{i}\right)\right\}. \end{array}$$

Therefore, the final output through the proposed model for an *N*-input neuron is obtained by equation (8) as follows:

(8) $$\begin{array}{c} O=\phi \left(v\right). \end{array}$$

Further simplifying the proposed model (as given by equation (7)), we have the following:

(9) $$\begin{array}{c} v={\left(-1\right)}^{N+1}\times b^{N}\times \prod_{i=1}^{N}\left(x_{i}+t_{i}\right). \end{array}$$

### 5.1. Scaling Factor in Proposed Model

The issue of vanishing gradient and nonconvergence in the previous *π*_*t*_-neuron model has been resolved by our proposed neuron model. It is because of the input dimension-dependent adaptable scaling factor (given in equation (6)). The effect of the scaling factor is already discussed in the previous section (as depicted in Figure 2(b)). We have seen that a larger scaling factor supports BP and results from proper convergence in the case of higher dimensional input. The significance of scaling has already been demonstrated in Figure 2(b).  Figure 4 is the demonstration of the optimal value of scaling factor ‘*b*'.

To illustrate the significance of the optimized value of scaling factor ‘*b*', we have plotted the gradient of sigmoid function ‘*ϕ*ʹ(*x*)' by considering variation in the values of ‘*b*' in Figure 3. It is observed from the plot that the scaling factor, *b* = 1, has poor sensitivity for any change in the input. Also, the sensitivity of the ‘*ϕ*ʹ(*x*)' increases by increasing the value of scaling factor ‘*b*'. However, as we increase the scaling factor ‘*b*' more than 6, we have poor sensitivity regions again, causing gradient vanishing problems. Vanishing gradient regions are shown by encircled areas in the plot. It shows an optimal value is between (3 ∼ 6). For less than three, it has smaller sensitivity, and for more than six, it again shows the gradients vanishing problem. In our experiment, we have empirically found that initializing the scaling factor ‘*b*' with the value ‘4' for each input results in successful training. However, we require to fine-tune the scaling factor according to the input and its dimension.

Therefore, we have considered the optimization of the scaling factor depending on the dimension and value of the input in our model. Therefore, we have considered an adaptable scaling factor (*b*_*i*_) which is associated with each input (*x*_*i*_) in our proposed model (as given by Equation (6)). Further, it has another advantage in that it helps in rapidly achieving the optimized value of the scaling factor without changing the learning rate in training the model. It eventually helps in achieving convergence using the BP algorithm in training the model. Mathematically, the error gradient (∇*Ɛ*) associated with our proposed neuron model (obtained by equations (3)–(5)) is defined as follows:

(10) $$\begin{array}{c} \frac{\partial \varepsilon \left(n\right)}{\partial b\left(n\right)}=\delta \left(n\right)\times \text{N}\times b^{N-1}\times \prod \left(x_{k}\left(n\right)+t_{k}\left(n\right)\right),\\ \frac{\partial \varepsilon \left(n\right)}{\partial t_{i}\left(n\right)}=\delta \left(n\right)\times b^{N}\times \prod \left(x_{k}\left(n\right)+\;t_{k}\left(n\right)\right);\forall \left(i\neq k\right). \end{array}$$

Here, the larger scaling factor ‘*b*^*N*^' accurately compensates for infinitesimally small gradient problems. Therefore, the larger scaling factor enforces a sharper transition to the sigmoid function and supports easier learning in case of higher dimensional parity problems. In the proposed model, the scaling factor is trainable and depends upon the number of input bits. It has exponent term as the no. of input bits means, for higher input we have sharper transition which compensates for infinitesimally small gradient problems. Therefore, the proposed enhanced *π*_*t*_-neuron model has no limitation for higher dimensional inputs.

### 5.2. Sign-Manipulation in the Proposed Model

The enhanced *π*_*t*_-neuron is based on the multiplicative neuron model. The multiplicative model suffers from a class reversal problem. It is the reversal of class depending upon the number of input bits. It is because of the sign change property of the multiplicative model according to even and odd input dimensions. This leads to severe confusion in classification. To mitigate this issue, we have multiplied a sign-manipulation factor as ‘(‒1)^*N+1*^'. Therefore, it introduces an extra negative sign for the even number of input bits to maintain the input combinations belonging to the same class. These two (scaling factor and sign-manipulation) modifications in the existing *π*_*t*_-neuron model have enhanced its performance for highly dense XOR data distribution and higher-order *N*-bit parity problems.

## 6. Results and Discussion

We have used gradient–decedent algorithm for training the proposed neuron model. The binary cross-entropy loss function is used for estimating loss between target and trained threshold vectors training on a single ‘*Nvidia Geforce eXtreme 1080*' graphic card. The efficacy of the proposed neuron has been evaluated for generalized XOR problems. We have considered a typical highly dense two-input XOR data distribution, as shown in Figure 5. It is applied to both models (i.e., the *π*_*t*_-neuron model and the proposed model) to compare the efficacy of the model. There are many popular loss functions to visualize the deviation in desired and predicted values, such as L_1_ loss, L_2_ loss, and L_∞_ loss. However, in our situation, data points vary between [0, 1], and L_1_ loss renders the best visualization in such cases. Therefore, we have considered the L_1_ Loss function, which is the least absolute deviation, and used it to estimate the error. The L_1_ loss (ℒ) is defined as follows:

(11) $$\begin{array}{c} ℒ=\sum_{i=1}^{N}\left|{\left(\text{desired}\right)}_{i}-{\left(\text{predicted}\right)}_{i}\right|. \end{array}$$

Since random weights and biases are important in the training of the model. That is why we have considered He-initialization [36] in our approach. It is a variant of Xavier-Initialization [37]. In He-initialization, the biases are initialized with 0.0 (zero value) and the weight is initialized using Gaussian probability distribution (*G*) given as $\left(W\right)∼G\left(0,\sqrt{2/r_{l}}\right)$ for ‘*l*^*th*^' layer. Here, ‘*r*' denotes the number of connections. Further, to assess the applicability and generalization of our proposed single neuron model, we have varied the input dimension and no. of input samples in training the proposed model. We have considered three different cases having 10^3^, 10^4^, and 10^6^ samples in the dataset, respectively. Results (in all three cases) have been summarized in Table 2. Results show that the loss depends upon the no. of samples in the dataset. It decreases by increasing the number of samples.

Number of samples required in the XOR dataset for appropriate training depends upon the input dimension. It is given by the following equation:

(12) $$\begin{array}{c} p=2^{N}. \end{array}$$

Here, ‘*p*' is the number of required samples for ‘*N*' dimensional input. To understand this relation, consider two-dimensional datasets (i.e., *N* = 2). Therefore, the no. of the required sample (i.e., *p*) is obtained by (9) as (*p* *=* *2*^*2*^ = 4). It is the classical exclusive OR (XOR) dataset, represented as {(0, 0), (0, 1), (1, 0), (1, 1)}. Similarly, if (*N* = 3), then (*p* *=* *2*^*3*^ = 8), which indicates a three-input XOR dataset, and so on. Lesser samples in the training dataset cause nonconvergence and inaccuracy.

Equation (12) tells the number of samples required in the training dataset. Therefore, for ten-dimensional input, the number of samples required for training should be (*p* *=* *2*^*10*^ = 1024). Therefore, approximately 1,000 samples are sufficient for a ten-dimensional training dataset. However, if we increase the dimension, it requires more no. of samples to train the model appropriately. Otherwise model fails to get converge. The same is shown in Table 3. To assess the accuracy of our proposed model, we repeated each experiment 25 times and provided accurate results. Here, the success rate signifies the ratio of successful simulation over total simulations for each case. In the case of ten-dimensional input for 1000 training samples, the success rate is 0.96, whereas it is reduced to 0.76 in the case of thirteen-dimensional input because of insufficient training samples. However, if we increase the no. of training samples to 10,000, the model report 100% of success ratio. Similarly, for 20 bits input (*p* *=* *2*^*20*^ = 1,048,576), samples are required. Therefore, by training 1,000 samples, the success ratio is 0.0, while for 10,000 samples, it is 0.32. It increases further to 0.64 for one million samples. These results furnish the importance of no. of training samples for solving XOR type nonlinear problems. Also, by observing the results, we can easily understand the capability of the proposed model for generalized XOR type real problems.

Further, the proposed algorithm has been repeated 30 times to assess the performance of its training. The standard statistical indicators such as mean (*μ*) and standard deviation (*σ*) are considered the assessment parameters of the predicted values.  Table 4 provides the prediction results (in terms of threshold values (*t*_*1*_, *t*_*2*_) and scaling factor (*b*)) obtained by the proposed models. It also showcases the mean and standard deviations of the predicted thresholds and bias values.

Table 5 provide values of the threshold obtained by both the *p*_t_-neuron model and proposed models. In experiment #2 and experiment #3, the *p*_t_-neuron model has predicted threshold values beyond the range of inputs, i.e., [0, 1]. This is because we have not placed any limit on the values of the trainable parameter. It only reflects that the *π*_*t*_-neuron model has been unable to obtain the desired value in these experiments.

L_1_ loss (ℒ) obtained in these three experiments for the *π*_*t*_-neuron model, and the proposed model is provided in Table 3. This loss function is only used to visualize the comparison in the model. As mentioned earlier, we have used the binary cross-entropy loss function to train our model.

It is observed by the results of Tables 5 and 6 that the *π*_*t*_*-*neuron model has a problem in learning highly dense XOR data distribution. However, the proposed neuron model has shown accurate classification results in each of these cases. Also, the loss function discerns heavy deviation as predicted and desired values of the *π*_*t*_-neuron model.

Further, we have monitored the training process for both models by measuring the binary cross-entropy (BCE) loss versus the number of iterations (as shown in Figure 6). We should remember that it is the cross-entropy loss on a logarithmic scale and not the absolute loss. It supports backpropagation error calculation which is an issue with smaller errors. It is generally considered an appropriate loss metric in classification problems. Therefore, we have used BCE as a measure to observe the trend of training to compare the *π*_*t*_-neuron model with our proposed model. As observed, the proposed model has achieved convergence which is not obtained by the *π*_*t*_-neuron model. We have examined the performance of our proposed model over *N*-bit parity problems. We have considered similar data distribution (as that in Figure 5) for parity problems as well. Further, we have compared the training performance of the *π*_*t*_-neuron model with our proposed model for the 10-bit parity problem. Training results of both models have been represented in Figure 7 (by plotting binary cross-entropy loss versus the number of iterations).

We have examined the performance of our proposed model for higher dimensional parity problems. It is to assess the applicability and generalization of our model. We have randomly varied the input dimension from 2 to 25 and compared the performance of our model with *π*_*t*_-neuron. Results are tabulated below.  Table 7 provides the scaling factor and loss obtained by both *π*_t_-neuron and proposed neuron models.

As mentioned earlier, we have measured the performance for the *N*-bit parity problem by randomly varying the input dimension from 2 to 25. L_1_ loss function has been considered to visualize the deviations in the predicted and desired values in each case. The proposed model has shown much smaller loss values than that of with *π*_*t*_-neuron model. Also, the proposed model has easily obtained the optimized value of the scaling factor in each case. Tessellation surfaces formed by the *π*_*t*_-neuron model and the proposed model have been compared in Figure 8 to compare the effectiveness of the models (considering two-dimensional input).

This is observed here that the proposed model has formed an enhanced tessellation surface than that of the *π*_*t*_-neuron model. It is merely because of the optimal scaling. In the case of the *π*_*t*_-neuron model, the scaling factor is (*b*_*π‒t*_ = ‒1.7045), whereas our model has obtained the scaling factor as (*b* = 4.6900). As we have discussed earlier, the value of the scaling factor associated with input should be around (4) for each input (described in Figure 4). Further, because of the two-dimensional problem, the effective scaling factor in our case is (*b*^*N*^ = 21.9961). We have plotted the effective values of the scaling factor in our proposed model and the *π*_*t*_-neuron model on a logarithmic scale to visualize the effect of scaling with increasing input dimension in Figure 9.

The trend of variation of the effective scaling factor with an increasing dimension of input discerns that the proposed model can rapidly increase the required value of the scaling factor to compensate for the effect of miniaturization of errors within higher dimensional input. However, the previous *π*_*t*_-neuron model has no such ability. This is possible in our model by providing the compensation to each input (as given in our proposed enhanced *π*_*t*_-neuron model by equation (6)). We have considered the input distribution similar to Figure 5 (i.e., the input varies between [0, 1]) for each dimension. Results show that the effective scaling factor depends upon the dimension of input as well as the magnitude of the input. Therefore, our proposed model has overcome the limitations of the previous *π*_*t*_-neuron model.

Further, the computational complexity of the proposed model is obtained from the investigation of Schmitt in [38]. Schmitt has investigated the computational complexity of multiplicative neuron models. They have used the Vapnik-Chervonenkis (VC) dimension and the pseudo dimension to analyze the computational complexity of the multiplicative neuron models. The VC dimension is a theoretical tool that quantifies the computational complexity of neuron models. According to their investigation for a single product unit the VC dimension of a product unit with *N*-input variables is equal to *N*.

## 7. Discussion and Conclusions

Translated multiplicative (*π*_*t*_) neuron model has been suggested by past researchers to solve the XOR and *N*-bit parity problems. However, it has an issue in backpropagation for densely distributed XOR and higher dimensional parity problems. It is an indigenous problem associated with multiplicative neuron models. Though the *π*_*t*_-neuron model has a scaling factor in subduing this problem, however, without suitable initialization, it is unable to obtain the appropriate scaling factor for higher-dimensional input. Therefore, a generalized solution is still required to overcome these issues. In this paper, an enhanced translated multiplicative neuron modeling has been proposed to enhance the performance of the *π*_*t*_-neuron model. The proposed model can obtain the optimized value of the scaling factor for any input dimension. It has solved the existing backpropagation issue of the *π*_*t*_-neuron model. We have considered an adaptable scaling factor associated with each input in our proposed model. This helps in achieving optimal scaling factor value for higher dimensional input. We have assessed the efficacy of our model by randomly increasing input dimensions and considered a magnitude variation between [0, 1] for each input. The proposed model has outperformed the *π*_*t*_-neuron model in each case. It has shown more than an 80% reduction in absolute loss as compared to the previous neuron model in similar experimental conditions. Also, the proposed model has formed a more accurate tessellation surface as compared to the previous model for two-dimensional input. Further, there are multiple real-world implementations involving the time series forecasting and classification such as trends analysis, seasonal (weather) predictions, cycle, and irregularity predictions. These real-world problems are associated with forecasting and classifications of time-series data. A multiplicative neuron model is commonly employed in such predictions and renders superior results. Our proposed single multiplicative neuron model has overcome the limitations of dimensionalities. Therefore, it can be easily employed in such prediction tasks as well.

## Figures and Tables

**Figure 1:** XOR problem is illustrated by considering each input as one dimension and mapping the digital digit ‘*0*' as negative axis and ‘*1*' as the positive axis. Therefore, XOR data distribution is the areas formed by two of the axes ‘*X*_*1*_' and ‘*X*_*2*_', such that the negative area corresponds to class *1*, and the positive area corresponds to class *2*.

**Figure 2:** (a) Sigmoid function *ϕ(x)*; (b) effect of scaling on *ϕ(x)*.

**Figure 3:** Proposed translated multiplicative neuron architecture.

**Figure 4:** Effect of scaling factor on the gradient of the sigmoid function.

**Figure 5:** A typical highly dense two-input XOR data distribution.

**Figure 6:** Training progress of both models (i.e., *π*_*t*_-neuron model and proposed model). Here, we have considered a typical highly dense two-input XOR data distribution. The result shows that the *π*_*t*_-neuron model has an issue in training while the proposed model has achieved convergence.

**Figure 7:** Results show the training progress of both models (i.e., *π*_*t*_-neuron model and proposed model) for the 10-bit parity problem. The proposed model has achieved convergence while the *π*_*t*_-neuron model has not.

**Figure 8:** Tessellation surface formed by *π*_*t*_*-*neuron model and proposed model for two-dimensional input.

**Figure 9:** Trend of scaling factor variation for (N)-bit parity problem is compared in both of the models (i.e., *π*_*t*_*-*neuron model and proposed model). Here, the effective scaling factor for a *π*_*t*_-neuron model is ‘(*b*_*π‒t*_)', whereas for the proposed model ‘*b*^*N*^.'

**Table 1:** List of variables used in this article with their meaning.

Variables	Meaning
*π*-neuron	Multiplicative neuron model
*π*_t_-neuron	Symbol of translated multiplicative neuron model
Π	Product operator
*v*_*π*‒t_	The mathematical form of the *p*_t_-neuron model
*f*	Activation function
*x*_*i*_	‘*i*^*th*^' input to the neuron
y	The final output of the *p*_t_-neuron model through the activation function ‘*f*'
*b*_*π‒t*_	Scaling factor associated with the *p*_t_-neuron model
*t*_*i*_	The coordinates of the center of the decision surfaces (‘*i*^*th*^' threshold value)
*δ*(*n*)	The local gradient in the backpropagation algorithm at ‘*n*^*th*^' iteration
*ϕ*(*x*)	Sigmoid activation function
*Ɛ*(*n*)	The error energy (the instantaneous sum of the error squares at ‘*n*^*th*^' iteration)
*∇Ɛ*	Error gradient
*e*(*n*)	The error value in the backpropagation algorithm at ‘*n*^*th*^' iteration
*ϕ′*	Derivative of the sigmoid activation function
*b*	Scaling factor associated with the enhanced *p*_t_-neuron model (proposed)
*v*	The mathematical form of the proposed model
*O*	The final output of the proposed model through the activation function ‘*ϕ*'
*ℝ*	Set of the real numbers
*L*_*1*_, *L*_*2*_, *L*_*∞*_	Respective loss functions
*ℒ*	L_1_ loss function
*W*	Weight matrix
*G*	Gaussian probability distribution
*p*	Number of samples required in an XOR dataset for appropriate training
*μ*	Mean or average value
*σ*	Standard deviation value

**Table 2:** Assessment of Proposed Model (through variation in dimension and no. of training samples).

Dimension (*N*)	10^3^		10^4^		10^6^	
	*Time* (*s*)	ℒ (*Ours*)	*Time* (*s*)	ℒ (*Ours*)	*Time* (*s*)	ℒ (*Ours*)
2	0.710	0.0195	0.712	0.0195	1.571	0.0244
5	0.692	0.0105	0.768	0.0091	2.808	0.0088
7	0.686	0.0093	0.759	0.0064	3.822	0.0058
10	0.688	0.0184	0.770	0.0048	5.806	0.0040
13	0.693	0.0577	0.790	0.0045	7.666	0.0023
15	0.703	0.2156	0.793	0.0126	9.435	0.0020
18	0.696	0.9041	0.805	0.1501	8.497	0.0150
20	0.701	0.9883	0.812	0.2441	9.378	0.0679
25	0.701	1.2155	0.811	0.3790	11.982	0.1188

**Table 3:** Success Rate (through variation in dimension and no. of training samples).

Dimension (*N*)	10^3^	10^4^	10^6^
2	1.0	1.0	1.0
5	1.0	1.0	1.0
7	1.0	1.0	1.0
10	0.96	1.0	1.0
13	0.76	1.0	1.0
15	0.32	0.96	1.0
18	0.0	0.40	0.92
20	0.0	0.32	0.64
25	0.0	0.0	0.24

**Table 4:** Predictions Through the Proposed Model (in terms of threshold values (*t*_*1*_, *t*_*2*_), and scaling factor (*b*)).

Experiment no.	*t*_*1*_	*t*_*2*_	*b*
1	0.4982	0.5097	3.9651
2	0.5049	0.5079	3.97
3	0.4958	0.5113	3.9869
4	0.5099	0.4967	3.98
5	0.5015	0.4967	3.969
6	0.4903	0.5014	3.9693
7	0.5002	0.5076	3.9652
8	0.504	0.511	3.9638
9	0.4973	0.5138	3.9872
10	0.4995	0.4887	3.9773
11	0.5031	0.497	3.9777
12	0.4945	0.497	3.9802
13	0.5019	0.4989	3.9773
14	0.4974	0.4895	3.9688
15	0.4921	0.5024	3.9807
16	0.4943	0.5106	3.9858
17	0.5074	0.5101	3.9697
18	0.5075	0.4975	3.9686
19	0.4914	0.4959	3.9702
20	0.4974	0.4888	3.9772
21	0.5019	0.5138	3.9628
22	0.5084	0.5005	3.9631
23	0.5085	0.5055	3.964
24	0.5138	0.4993	3.9742
25	0.5063	0.5026	3.9634
26	0.5022	0.4901	3.9702
27	0.503	0.5147	3.9866
28	0.4992	0.4831	3.9636
29	0.512	0.4983	3.9696
30	0.4968	0.4975	3.9706
Mean (*μ*)	0.5014	0.5013	3.9726
Standard deviation (*σ*)	0.00614	0.00849	0.00781

**Table 5:** Comparison of Π_*t*_-Neuron Model and Proposed Model (in terms of threshold values).

Experiment no.	Desired		Predicted (*p*_t_)		Predicted (ours)	
	*t*_*1*_	*t*_*2*_	*t*_*1*_	*t*_*2*_	*t*_*1*_	*t*_*2*_
1	0.5	0.5	0.6023	0.1546	0.5024	0.5037
2	0.580	0.672	0.5567	2.6124	0.579	0.674
3	0.460	0.084	0.4679	‒15.9951	0.459	0.085

**Table 6:** L_1_ loss (ℒ) Obtained by Π_*t*_-Neuron Model and Proposed Model.

Experiment no.	ℒ (*π*_*t*_)	ℒ (Ours)
1	0.1744	0.003
2	0.9818	0.0015
3	8.0435	0.001

**Table 7:** Scaling Factor and loss Obtained by Π_t_-Neuron and Proposed Models with Increasing Input Dimension of *N*-bit Parity Problem.

*N*	Scaling factor		L_1_ loss (ℒ)	
	*π*_*t*_-neuron (*b*_*π‒t*_)	Ours (*b*)	*π*_*t*_-neuron	Ours
2	‒1.7045	4.6900	0.3281	0.0093
5	0.3911	4.2760	2.1059	0.0093
7	72.1092	4.2208	0.8367	0.0058
10	‒42.6576	4.0720	0.5690	0.0047
13	33.9146	4.0548	1.0349	0.0037
15	64.4870	3.9516	0.8966	0.0079
18	‒20.1572	3.8317	0.9393	0.0072
20	‒79.3860	3.9426	0.8311	0.0072
25	83.9456	3.7275	0.9855	0.1431

## Data Availability

The data used to support the findings of this study are included in the article.

## References

[1] Minsky M. L., Perceptrons S. A. P.. (2017). *An Introduction to Computational Geometry*.

[2] Amir H. E., Hamdy M. (2020). Deep learning fundamentals. *Deep Learning Pipeline*.

[3] Özdemir A., İnal M. M. (2016). Only one neuron either N-bit parity rule based modified translated multiplicative or McCulloch-pitts models for some machine learning problems. *International Journal of Intelligent Systems and Applications in Engineering*.

[4] Rosen B. E., Goodwin J. M., Vidal J. J. Transcendental functions in backward error propagation.

[5] Kaveh A., Vogh J. Influence of different nonlinearity functions on Perceptron performance.

[6] Zhang Z., Sarhadi M. A modified neuron activation function which enables single layer perceptrons to solve some linearly inseparable problems.

[7] Labib R. New single neuron structure for solving nonlinear problems.

[8] Wu Y., Zhao M., Ding X. (1997). A new kind of neuron model with a tunable activation function and its applications. *Science in China - Series E: Technological Sciences*.

[9] Wu Y., Zhao M. (2001). A neuron model with trainable activation function (TAF) and its MFNN supervised learning. *Science in China, Series A: Information Sciences*.

[10] Yanling Z., Bimin D., Zhanrong W. Analysis and study of perceptron to solve XOR problem.

[11] Nitta T. (2003). Solving the XOR problem and the detection of symmetry using a single complex-valued neuron. *Neural Networks*.

[12] Shen Y., Wang B., Chen F., Cheng L. (2004). A new multi-output neural model with tunable activation function and its applications. *Neural Processing Letters*.

[13] Amin M. F., Murase K. (2009). Single-layered complex-valued neural network for real-valued classification problems. *Neurocomputing*.

[14] Tsapanos N., Tefas A., Nikolaidis N., Pitas I. (2018). Neurons with paraboloid decision boundaries for improved neural network classification performance. *IEEE Transactions on Neural Networks and Learning Systems*.

[15] Sagheer A., Zidan M., Abdelsamea M. M. (2019). A novel autonomous perceptron model for pattern classification applications. *Entropy*.

[16] Iyoda E. M., Nobuhara H., Hirota K. (2003). A solution for the *N*-bit parity problem using a single translated multiplicative neuron. *Neural Processing Letters*.

[17] Iyoda E. M., Nobuhara H., Hirota K. (Apr. 2004). Translated multiplicative neuron: an extended multiplicative neuron that can translate decision surfaces. *Journal of Advanced Computational Intelligence and Intelligent Informatics*.

[18] Bland R. (1998). *Learning XOR: Exploring the Space of a Classic Problem*.

[19] Durbin R., Rumelhart D. E. (1989). Product units: a computationally powerful and biologically plausible extension to backpropagation networks. *Neural Computation*.

[20] Leerink L. R., Giles C. L., Horne B. G., Jabri M. A. (1995). Learning with product units. *Advances in Neural Information Processing Systems*.

[21] Haykin S. (1999). Multilayer perceptrons. *Neural Networks: A Comprehensive Foundation*.

[22] Bakr M. H., Negm M. H. (2012). Modeling and design of high-frequency structures using artificial neural networks and space mapping. *Advances in Imaging and Electron Physics, *.

[23] Karlik B., Olgac A. V. (2011). Performance analysis of various activation functions in generalized MLP architectures of neural networks. *International Journal of Artificial Intelligence and Expert Systems*.

[24] Yildirim A. N., Bas E., Egrioglu E. (2021). Threshold single multiplicative neuron artificial neural networks for nonlinear time series forecasting. *Journal of Applied Statistics*.

[25] Yolcu O. C., Bas E., Egrioglu E., Yolcu U. (2018). Single multiplicative neuron model artificial neural network with autoregressive coefficient for time series modelling. *Neural Processing Letters*.

[26] Egrioglu E., Yolcu U., Aladag C. H., Bas E. (2015). Recurrent multiplicative neuron model artificial neural network for nonlinear time series forecasting. *Neural Processing Letters*.

[27] Yadav R. N., Kalra P. K., John J. (2007). Time series prediction with single multiplicative neuron model. *Applied Soft Computing*.

[28] Pan W., Zhang L., Shen C. (2021). Data-driven time series prediction based on multiplicative neuron model artificial neuron network. *Applied Soft Computing*.

[29] Egrioglu E., Bas E. (2022). A new automatic forecasting method based on a new input significancy test of a single multiplicative neuron model artificial neural network. *Network: Computation in Neural Systems*.

[30] Gao S., Zhou M., Wang Y., Cheng J., Yachi H., Wang J. (2018). Dendritic neuron model with effective learning algorithms for classification, approximation, and prediction. *IEEE Transactions on Neural Networks and Learning Systems*.

[31] Zhang Z. H., Min F., Chen G. S., Shen S. P., Wen Z. C., Zhou X. B. (2021). Tri-partition state alphabet-based sequential pattern for multivariate time series. *Cognitive Computation*.

[32] Ran X., Zhou X., Lei M., Tepsan W., Deng W. (2021). A novel k-means clustering algorithm with a noise algorithm for capturing urban hotspots. *Applied Sciences*.

[33] Cui H., Guan Y., Chen H., Deng W. (2021). A novel advancing signal processing method based on coupled multi-stable stochastic resonance for fault detection. *Applied Sciences*.

[34] Deng W., Zhang X., Zhou X. (2022). An enhanced fast non-dominated solution sorting genetic algorithm for multi-objective problems. *Information Sciences*.

[35] Wu E. Q., Zhou M., Hu D. (2020). Self-paced dynamic infinite mixture model for fatigue evaluation of pilots’ brains. *IEEE Transactions on Cybernetics*.

[36] He K., Zhang X., Ren S., Sun J. Delving deep into rectifiers: surpassing human-level performance on imagenet classification.

[37] Glorot X., Bengio Y. Understanding the difficulty of training deep feedforward neural networks.

[38] Schmitt M. (2002). On the complexity of computing and learning with multiplicative neural networks. *Neural Computation*.

